# Detection Scheme for Tampering Behavior on Distributed Controller of Electric-Thermal Integrated Energy System Based on Relation Network

**DOI:** 10.1155/2022/9594267

**Published:** 2022-08-27

**Authors:** Chaoqun Zhu, Jie Li, Jie Shen, Lei Zhou, Xiaoming Zhang, Dan Zhu, Yafei Li

**Affiliations:** Marketing Department of State Grid Suzhou Power Supply Company, Suzhou 215000, China

## Abstract

In recent years, with the development of smart grid, the power systems and other energy systems are gradually forming integrated energy systems. The electric-thermal integrated energy system is a mature integrated energy system at present. The electric-thermal integrated energy system uses modern communication technology to realize the comprehensive regulation of electric energy and thermal energy, which greatly improves the efficiency of energy use. However, this also greatly increases the risk of malicious tampering with the energy dispatch system. In this paper, we study the regulation of electric-thermal integrated energy systems considering false data injection attacks. First, we establish a compromised model of an electric-thermal integrated energy system considering false data injection attacks. Then, we designed vulnerable variable observers for different tampering scenarios to observe the tampered variables. Finally, considering the relationship between the observed data and the measured data, we design a tampering behavior detection method based on relation network. The simulation results verify the effectiveness of the detection method proposed in this paper.

## 1. Introduction

The electric-thermal integrated energy system (ETIES) is an important part of the integrated energy system. With the aid of the advanced network information technology and innovative operation and management models, ETIES integrates electrical and thermal energy in the region, realizes operation optimization and coordinated control among various heterogeneous energy sub-networks through energy coupling equipment, and effectively improves energy conversion efficiency and promotes sustainable energy while meeting the diverse energy needs of users [1–3]. However, ETIES based on distributed optimization architecture is a highly integrated information-physical energy system. The information system of ETIES is bound to endure a huge threat of cyber attacks while exchanging a large amount of information data [4, 5].

The spread of malicious attacks in the communication network will destroy the environment of network communication, make the economic operation of the system impossible, even destroy the stability of the system [6, 7]. In [8], the authors propose that the measurement equipment in the cyber physical system suffer from multiple types of cyber-attacks, and summarizes the current mainstream attack defense schemes based on learning-based methods. In [9], the authors propose that the energy-water nexus with multiple sensors may be vulnerable to cyber-attacks. To deal with the potential threats, an observer-based attack detection method is proposed. As a typical information-physical system, the monitoring and control of power system highly depends on the accuracy of measured data [10]. When the measurement data is compromised, the operation stability and security of the power system will be greatly reduced, thus threatening social security and social economy. To enhance the resilience of the sensors in power systems, the attack defense scheme based on the features of the measured data is proposed. This type of attack detection scheme enables cyber physical system to maintain good detection performance under cyber-attacks.

False data injection attack (FDI attack) is a new form of attack that has appeared in recent years to undermine the credibility of the operational data of integrated energy systems [11, 12]. When the attacker has the ability to inject data streams into the data transmission channel of the integrated energy system, attack vectors can be constructed targeting the vulnerabilities of the traditional bad data detection methods and identification methods of the integrated energy system, and arbitrarily manipulate the data of the attacked data channel of the integrated energy system. The flow changes the real data of the system into false data, which affects the real-time operation status of the power system, thus threatening the stable, safe and economic operation of the power system. Therefore, it is necessary to improve the attack defense capability of monitoring node sensors to resist the damage to the system caused by cyber-attacks [13, 14].

At present, there are two main perspectives in the research on considering the existence of FDI attacks in the system. On the one hand, from the perspective of FDI attackers, researchers design an optimal attack strategy that can improve the probability of successful attack and attack effect. Reference [15] studies the attack vector construction method from the attacker's point of view. Combining the *l*_0_ norm and *l*_1_ norm of the attack vector, an attack evaluation index to measure the attack effect and attack cost is proposed. References [16–18] considered the scenarios where the measurement data in the actual system has different security protection levels, and proposed a corresponding minimum attack vector construction method. In order to reduce the attack cost and improve the attack efficiency, the literature [19, 20] designed an attack vector construction method based on the minimum cut set with the goal of making the energy system lose its ability to observe the external environment. At the same time, other attack scenarios can also be considered when constructing false data injection attack vectors. The attacker in [21] used traditional attack methods such as worms to break through the firewall and obtained the control authority of the basic equipment, and then launched a false data injection attack to tamper with the state variables of the energy system, thereby causing cascading failures of associated equipment. Reference [22] proposed a form of attack based on false data injection attacks to attack the topology of power systems—Man-in-the-middle attacks (MITM attacks). In this form of attack, the attacker eavesdrops on the data transmission terminals of the power system, and spoofs the status of the power system equipment by injecting false data. At this time, the communication mode between data transmission terminals changes from direct communication in normal state to relay communication through third-party devices, and the reliability of the association state between devices will be destroyed. Reference [23] demonstrates the attack effect of a multi-level MITM attack with the help of a simulation platform. The simulation results show that this type of attack can mislead the control center to make a wrong assessment of the current energy system topology by controlling the switch state between the devices, and trigger misoperations to cause power system physical layer accidents. Reference [24] added a data frame attack to the man-in-the-middle attack based on the normalized residual search method. Different from traditional false data injection attacks, which aim to maintain the concealment of false data, the main purpose of this type of attack is to deliberately launch bad data detection (BDD) to make real data be regarded as false data, thereby disturbing state estimation of energy system.

On the other hand, researchers propose defense strategies against network attacks from the perspective of system defense. References [25, 26] use Petri nets to describe the information flow between data interaction terminals in a power cyber-physical system and propose a cooperative intrusion detection algorithm against false data injection attacks. The analysis model based on Petri net can clearly describe the transient and steady-state reliability of power system under multiple attack events. The detection of false data injection attacks based on machine learning algorithms is also a research direction that domestic and foreign researchers focus on. Reference [27] considered the behavior characteristics of false data injection attacks against load frequency control systems, and designed an intelligent attack detection algorithm based on multi-layer perceptrons to effectively identify false data injection attacks. Reference [28] considered the behavior characteristics of false data injection attack on power system transmission lines, using programmable logic controller as a detection method. The computing node of the algorithm is tested, and the classifier of machine learning is used to realize the identification of false data injection attacks. This distributed attack detection algorithm can effectively reduce decision-making delay and improve attack detection efficiency. Reference [29] proposed an unsupervised attack detection scheme based on the isolation forest algorithm, and used the principal component analysis method to extract the features of the power system variables, thereby reducing the dimensionality problem in the machine learning process. Reference [30] considered the problem of a small number of abnormal samples in the process of machine learning training, and proposed an intelligent attack detection algorithm using the support vector description domain to detect false data injection attacks in the load frequency control system. Reference [31] considered the false data injection attack form for load forecasting, proposed a machine learning-based load forecasting anomaly detection method, and estimated the false data injection attack type through naive Bayesian classification.

Similar to the original social power supply, heating and other systems, in the operation process of ETIES, one of the most concerned issues is how to realize the economic scheduling of the system, that is, how to comprehensively allocate the capacity distribution between multiple energy units on the premise of meeting the system security constraints, so as to minimize the economic cost of the system, and then realize the dual guarantee of system operation in terms of security and economy. The economic scheduling method of ETIES can be divided into centralized method and distributed method. Although the centralized method has high efficiency in information processing, it has some problems, such as high communication cost and sensitivity to single point of failure. The distributed method can use the sparse communication network structure to realize the decentralized cooperation of various equipment components of the system, which has less communication burden, stronger robustness and privacy. Therefore, in recent years, experts and scholars at home and abroad have proposed many ETIES economic scheduling methods based on distributed optimization.

However, it is worth noting that although the above method can effectively solve the distributed economic scheduling problem of ETIES, its premise is that the system operates in an ideal network communication environment, that is, a large number of interactive measurement and control data can be reliably transmitted on the communication line. However, ETIES based on distributed optimization architecture is an energy system with high integration of information and physics. While the information system of ETIES interacts with a large amount of information and data, it is bound to suffer from a huge threat of network attack. The spread of malicious attacks in the communication network will destroy the bad environment of network communication, make the economic operation of the system impossible, and even destroy the stability of the system, resulting in the paralysis of the energy supply system.

ETIES is a large system with electrical-thermal coupling characteristics, and its structure and operation are much more complex than traditional power systems. Therefore, malicious attackers need to adopt more complex and targeted strategies according to system conditions when attacking ETIES. So far, most of the research on the impact of network attacks on system performance is carried out on a single power system, and there is no research on the impact of network attacks on the operational security of ETIES. The distributed scheduling of ETIES depends on the security and reliability of the communication network, and network attacks will inevitably affect the scheduling process of ETIES, thereby affecting the performance of the system.

Aiming at this research gap, the motivation of the paper is to enhance the safety and security of the electric-thermal integrated energy system by studying the ETIES model under FDI attacks and designing an attack detection method based on machine learning algorithm.

The main contributions of the paper are three fold:

1. We establish attack templates in the electric-thermal integrated energy system and discuss the impact of false data injection attacks on the integrated energy system.
2. In the electric-thermal integrated energy system under FDI attack, we propose an observer-based method for observing vulnerable variables of the system, so that the compromised variables can be effectively observed.
3. Using the observation data obtained by the observer, we propose a relation network-based attack detection algorithm to detect FDI attacks in integrated energy systems.

The scope of the paper is shown as follows: first, the compromised model of the electric-thermal integrated energy system is discussed in this paper; Then, based on the variables in the system, a machine-learning-based attack detection method is studied to identify the FDI attacks on ETIES.

The remaining part of this paper is organized as follows: in Section 2, the model of the compromised electric-thermal integrated energy system under FDI attacks is established. In Section 3, the observer of the vulnerable variables is designed. In Section 4, the attack detection method based on relation network is designed. In Section 5, simulations are designed and the results are discussed. In Section 6, conclusions are stated.

### 1.1. Indices and Variables

*x*_*p*_^*P*^: Incremental cost of power only device.

*x*_*p*_^*C*^: incremental cost of combined heat and power device.

*x*_*h*_^*C*^: thermal incremental cost of combined heat and power device.

*x*_*h*_^*H*^: thermal incremental cost of heat only device.

*u*_*p*_^*P*^: electric power mismatch of power only device.

*u*_*p*_^*C*^: electric power mismatch of combined heat and power device.

*u*_*h*_^*C*^: thermal power mismatch of combined heat and power device.

*u*_*h*_^*H*^: thermal power mismatch of heat only device.

*m*(*k*): attack vector.

*y*_*p*_^*P*^: electric output power of power only device.

*y*_*p*_^*C*^: electric output power of combined heat and power device.

*y*_*h*_^*C*^: thermal output power of combined heat and power device.

*y*_*h*_^*H*^: thermal output power of heat only device.

*x*: state vector of the system.

$\bar{x}$ : augmented state vector of the system.

$\hat{\bar{x}}$ : observation of augmented state vector.

*e*: estimation error.

*d*_*m*_: data vector in the measured data set.

*d*_*o*_: data vector in the observed data set.

ℱ(*d*_*m*_): feature vectors of measured data.

ℱ(*d*_*o*_): feature vectors of observed data.

*𝒫*_*i*_^*m*^: prototype of the measured data feature vector in class *i*.

*𝒫*_*i*_^*o*^: prototype of the observed data feature vector in class *i*.

*N*_*i*_^*m*^: number of samples in class *i* of measured data feature vectors.

*N*_*i*_^*o*^: number of samples in class *i* of observed data feature vectors.

*𝒞*: concatenation module in relation network.

ℛ: relation module in relation network.

*𝒮*: similarity score in relation network.

*L*_*m*_: objective function in relation network.

*l*_*m*_: labels for measured data.

*l*_*o*_: labels for observed data.

*MA*: evaluation index of accuracy.

*MD*: evaluation index of the probability of detecting correctly.

*MS*: evaluation index of success ratio.

*MI*: evaluation index of probability of identifying normal cases.

*MF*: trade off between *MD* and *MS*.

### 1.2. Abbreviations

ETIES: electric-thermal integrated energy system.

FDI: false data injection.

MITM: man-in-the-middle.

BDD: bad data detection.

DDCA: distributed energy double-consensus algorithm.

POD: power only device.

CHP: COMBINED heat and power.

RELU: rectified linear unit.

## 2. FDI Attacks against Compromised Electric-Thermal Integrated Energy System and Countermeasures

In this section, we propose the FDI attacks against electric-thermal integrated energy system and study the countermeasures by designing the attack detection scheme. First, we introduce the basics of the energy management control strategy of electric-thermal integrated energy system, and propose the compromised model as the first step to mitigate FDI attacks. Second, based on the compromised model, we design observers to detect the variables compromised by FDI attacks. Finally, based on the observed data obtained by the proposed observers and the measured data obtained by measurement in ETIES, we propose an attack detection method to identify the safety status of ETIES.

### 2.1. Basics of Compromised Electric-Thermal Integrated Energy System

The typical distributed energy management method of electric-thermal integrated energy system is to use distributed energy double-consensus algorithm (DDCA). DDCA employs two different consensus protocols. One of the consensus protocols is used to calculate the incremental cost corresponding to the optimal solution of the ETIES economic dispatch problem. Another consensus protocol aims to estimate the amount of electrical/thermal local power mismatch for coordinating device output. The two protocols of DDCA use different but strongly coupled consistency variables to calculate the electric/thermal incremental cost, electric/thermal output power and electric/thermal local power mismatch corresponding to the optimal solution of ETIES economic dispatching problem, so as to finally realize the distributed economic dispatching of ETIES. ETIES scheduling depends on the information exchange and local calculation between each unit and its neighbors. Each energy unit contains a distributed controller for operation.

The attacker can attack the incremental cost estimator and the output power decision of the energy unit in DDCA, thereby affecting the output power of the unit in the energy unit. Inspired by reference [32], the compromised incremental cost estimator and output power decision-maker studied in this paper can be written as

(1) $$\begin{array}{c} \left\{\begin{array}{c} x\left(k+1\right)=Ax\left(k\right)+Bu\left(k\right),\text{normal,}\\ x\left(k+1\right)=Ax\left(k\right)+Bu\left(k\right)+Mm\left(k\right),\text{compromised,} \end{array}\right. \end{array}$$

where

(2) $$\begin{array}{c} x={\left[\begin{array}{cccc} x_{p}^{P} & x_{p}^{C} & x_{h}^{C} & x_{h}^{H} \end{array}\right]}^{T},\\ u={\left[\begin{array}{cccc} u_{p}^{P} & u_{p}^{C} & u_{h}^{C} & u_{h}^{H} \end{array}\right]}^{T}, \end{array}$$

where *A* is the consistency algorithm update matrix in DDCA, which is determined by the adjacency relationship between the current energy unit and the surrounding energy unit; *B* is the algorithm convergence rate adjustment matrix in DDCA; *M* is the corresponding attack weight matrix.

The compromised output power decision-maker studied in this paper can be written as

(3) $$\begin{array}{c} \left\{\begin{array}{c} y\left(k\right)=Cx\left(k\right),\text{normal,}\\ y\left(k\right)=Cx\left(k\right)+Nm\left(k\right),\text{compromised,} \end{array}\right. \end{array}$$

where

(4) $$\begin{array}{c} y={\left[\begin{array}{cccc} y_{p}^{P} & y_{p}^{C} & y_{h}^{C} & y_{h}^{H} \end{array}\right]}^{T}, \end{array}$$

where *C* is the cost coefficient matrix; *N* is the corresponding attack weight matrix.

It can be learned that FDI attacks can change the power output of the energy unit by tampering with the state variables of different modules in the ETIES, which has an impact on the power balance of the integrated energy system. In the next section, observers for different attack intrusion locations are designed to observe the FDI attacks.

## 3. Design of Observers for Detecting Compromised Variables in ETIES

### 3.1. Observer Design of Incremental Cost Estimator under FDI Attacks

In this part, we focus on the observer for compromised incremental cost estimator. The compromised system ∑_*ice*_ can be expressed as

(5) $$\begin{array}{c} \left\{\begin{array}{c} x\left(k+1\right)=Ax\left(k\right)+Bu\left(k\right)+Mm\left(k\right),\\ y\left(k\right)=Cx\left(k\right). \end{array}\right. \end{array}$$

Taking the attack vector *m*(*k* − 1) at *k* − 1 time as an additional state, we can obtain the augmented state vector $\bar{x}\left(k\right)={\left[x\left(k\right)m\left(k-1\right)\right]}^{T}$. The following augmented system can be established

(6) $$\begin{array}{c} \left\{\begin{array}{c} \bar{E}\bar{x}\left(k+1\right)=\bar{A}\bar{x}\left(k\right)+\bar{B}u\left(k\right),\\ y\left(k\right)=\bar{C}\bar{x}\left(k\right), \end{array}\right. \end{array}$$

where

(7) $$\begin{array}{c} \bar{E}=\left[\begin{array}{cc} I_{n} & -M\\ 0 & 0 \end{array}\right],\\ \bar{A}=\left[\begin{array}{cc} A & 0\\ 0 & 0 \end{array}\right],\\ \bar{B}=\left[\begin{array}{c} B\\ 0 \end{array}\right],\\ \bar{C}={\left[\begin{array}{c} C\\ 0 \end{array}\right]}^{T}. \end{array}$$

The following observer of the augmented system is designed

(8) $$\begin{array}{c} \left\{\begin{array}{c} z\left(k+1\right)=R\bar{A}\hat{\bar{x}}\left(k\right)+R\bar{B}u\left(k\right)+L\left(y\left(k\right)-\bar{C}\hat{\bar{x}}\left(k\right)\right),\\ \hat{\bar{x}}\left(k\right)=z\left(k\right)+Ty\left(k\right), \end{array}\right. \end{array}$$

where *z* represents the state vector of the dynamic system (4); *R*, *L* and *T* are the gain matrices with appropriate dimensions.

**Theorem 1 .**

When the compromised system has a state observer in the form equation (5), it needs to meet the following requirements: (1) $R\bar{E}+T\bar{C}=I_{n+q}$; (2) There are symmetric positive definite matrices *P* and *W* satisfying

(9) $$\begin{array}{c} \left[\begin{array}{cc} -P & {\left(R\bar{A}\right)}^{T}P-{\bar{C}}^{T}W^{T}\\ {}* & -P \end{array}\right]<0. \end{array}$$

**Proof**

Proof. Consider nonsingular matrices *U* ∈ *ℝ*^(*n*+*q*)×(*n*+*q*)^ and *V* ∈ *ℝ*^(*n*+*q*)×(*n*+*q*)^ such that

(10) $$\begin{array}{c} U\bar{E}V=\left[\begin{array}{cc} I_{N} & 0\\ 0 & 0 \end{array}\right]. \end{array}$$

Based on Sylvester inequality, we can derive

(11) $$\begin{array}{c} \text{rank}\left[\begin{array}{cc} I_{n} & 0\\ 0 & 0\\ C & 0 \end{array}\right]\\ =\text{rank}\left\{\left[\begin{array}{cc} U & 0\\ 0 & I_{m} \end{array}\right]\left[\begin{array}{c} \bar{E}\\ \bar{C} \end{array}\right]V\right\}\\ =\text{rank}\left[\begin{array}{c} \bar{E}\\ \bar{C} \end{array}\right]\\ =n+q. \end{array}$$

Therefore, we can derive

(12) $$\begin{array}{c} \text{rank}\left[\begin{array}{cc} I_{N} & 0\\ C & 0 \end{array}\right]\\ =\text{rank}\left[\begin{array}{c} \bar{E}\\ \bar{C} \end{array}\right]\\ =n+q,\\ \text{rank}\left(U\bar{E}V+\bar{C}V\right)=\text{rank}\left[\begin{array}{cc} I_{N} & 0\\ C & 0 \end{array}\right]=n+q. \end{array}$$

When the matrix to be designed *R* is

(13) $$\begin{array}{c} R=V{\left(U\bar{E}V+CV\right)}^{-1}U. \end{array}$$

Then the matrix *R* is a nonsingular matrix. Let the matrix *T* be

(14) $$\begin{array}{c} T=V{\left(U\bar{E}V+CV\right)}^{-1}. \end{array}$$

There exists $R\bar{E}+T\bar{C}=I_{n+q}$. The relationship between matrix [*R*, *T*] and matrix ${\left[\bar{E}\bar{C}\right]}^{T}$ is satisfied

(15) $$\begin{array}{c} \left[\begin{array}{c} \bar{E}\\ \bar{C} \end{array}\right]\left[\begin{array}{cc} R & T \end{array}\right]\left[\begin{array}{c} \bar{E}\\ \bar{C} \end{array}\right]=\left[\begin{array}{c} \bar{E}\\ \bar{C} \end{array}\right]. \end{array}$$

Then according to Moore Penrose theorem, it can be seen that [*R*, *T*] is a kind of generalized inverse matrix of ${\left[\bar{E}\bar{C}\right]}^{T}$, and has

(16) $$\begin{array}{c} \left[\begin{array}{cc} R & T \end{array}\right]={\left[\begin{array}{c} \bar{E}\\ \bar{C} \end{array}\right]}^{†}+\Theta \left(I_{n+q+m}-\left[\begin{array}{c} \bar{E}\\ \bar{C} \end{array}\right]{\left[\begin{array}{c} \bar{E}\\ \bar{C} \end{array}\right]}^{†}\right). \end{array}$$

Among them, Θ ∈ *ℝ*^(*n*+*q*)×(*n*+*q*+*m*)^ is a freely selected matrix, and the main purpose of parameter selection is to make *R* a nonsingular matrix.

For the system estimation error, we can derive

(17) $$\begin{array}{c} e\left(k\right)=\bar{x}\left(k\right)-\bar{\dot{x}}\left(k\right). \end{array}$$

Thus

(18) $$\begin{array}{c} e\left(k+1\right)=\left(R\bar{E}+T\bar{C}\right)x\left(k+1\right)-z\left(k+1\right)-Ty\left(k+1\right)\\ =R\bar{E}x\left(k+1\right)-z\left(k+1\right)\\ =\left(R\bar{A}-L\bar{C}\right)e\left(k\right). \end{array}$$

Select the following Lyapunov function

(19) $$\begin{array}{c} V\left(k\right)=e^{T}\left(k\right)Pe\left(k\right),\;P>0. \end{array}$$

We can derive

(20) $$\begin{array}{c} \Delta V\left(k\right)=V\left(k+1\right)-V\left(k\right)\\ =e^{T}\left(k\right)\left[{\left(R\bar{A}-L\bar{C}\right)}^{T}P\left(R\bar{A}-L\bar{C}\right)-P\right]e\left(k\right). \end{array}$$

If there exists matrix P and matrix L satisfying

(21) $$\begin{array}{c} \left[\begin{array}{cc} -P & {\left(R\bar{A}-L\bar{C}\right)}^{T}P\\ P\left(R\bar{A}-L\bar{C}\right) & -P \end{array}\right]<0. \end{array}$$

Then according to Schur complement theorem and Lyapunov stability theory, it can be obtained that Δ*V*(*k*) < 0 and *e*(*k*) is convergent. Let *W*=*PL*, then inequality equation (21) is equivalent to inequality equation (9).

The proof is completed. It can be learned that the defender can observe the system variables through the observer proposed in this paper when the incremental cost estimator is compromised.

### 3.2. Observer Design of Output Power Decision-Maker under FDI Attacks

In this part, we focus on the observer for compromised output power decision-maker. The compromised system ∑_*opd*_ can be expressed as

(22) $$\begin{array}{c} \left\{\begin{array}{c} x\left(k+1\right)=Ax\left(k\right)+Bu\left(k\right),\\ y\left(k\right)=Cx\left(k\right)+Nm\left(k\right). \end{array}\right. \end{array}$$

Taking the attack vector *m*(*k*) as an additional state, we can obtain the augmented state vector $\bar{x}\left(k\right)={\left[x\left(k\right)m\left(k\right)\right]}^{T}$. The following augmented system can be established

(23) $$\begin{array}{c} \left\{\begin{array}{c} \bar{E}\bar{x}\left(k+1\right)=\bar{A}\bar{x}\left(k\right)+\bar{B}u\left(k\right),\\ y\left(k\right)=\bar{C}\bar{x}\left(k\right), \end{array}\right. \end{array}$$

where

(24) $$\begin{array}{c} \bar{E}=\left[\begin{array}{cc} I_{n} & 0\\ 0 & 0 \end{array}\right],\\ \bar{A}=\left[\begin{array}{cc} A & 0\\ 0 & 0 \end{array}\right],\\ \bar{B}=\left[\begin{array}{c} B\\ 0 \end{array}\right],\\ \bar{C}={\left[\begin{array}{c} C\\ N \end{array}\right]}^{T}. \end{array}$$

Similarly, for this augmented system, we can also construct an observer in the form of formula (8). Conditions for the existence of observer are stated in Theorem 1. Due to space limitation, the proof of the existence of the observer is not repeated in this subsection. It can be learned that the observer design method based on augmented system can be effectively applied to the situations where incremental cost estimator or output power decision-maker is compromised.

### 3.3. Observer Design in Situations of Multiple Modules being Compromised considering Uncertainties

In this part, multipoint FDI attacks are considered: the attacker can launch FDI attacks on incremental cost estimator and output power decision-maker simultaneously. The compromised system ∑_*s*_ can be expressed as

(25) $$\begin{array}{c} \left\{\begin{array}{c} x\left(k+1\right)=Ax\left(k\right)+Bu\left(k\right)+Mm\left(k\right)+E_{a}\omega_{a}\left(k\right),\\ y\left(k\right)=Cx\left(k\right)+Nm\left(k\right)+E_{s}\omega_{s}\left(k\right), \end{array}\right. \end{array}$$

where *ω*_*a*_(*k*) and *ω*_*s*_(*k*) are unknown input vectors caused by uncertainties of system; *E*_*a*_ and *E*_*s*_ are known constant coefficient matrices with appropriate dimensions. Taking the attack vector as an additional state, we can obtain the augmented state vector $\bar{x}\left(k\right)={\left[\begin{array}{cc} x\left(k\right) & m\left(k\right) \end{array}\right]}^{T}$. The following augmented system can be established

(26) $$\begin{array}{c} \left\{\begin{array}{c} \bar{x}\left(k+1\right)=\bar{A}\bar{x}\left(k\right)+\bar{B}u\left(k\right)+\bar{E_{a}}\omega_{a}\left(k\right)+Gm^{d}\left(k\right),\\ y\left(k\right)=\bar{C}\bar{x}\left(k\right)+E_{s}\omega_{s}\left(k\right),\\ m^{d}\left(k\right)=m\left(k+1\right)-m\left(k\right), \end{array}\right. \end{array}$$

where

(27) $$\begin{array}{c} \bar{A}=\left[\begin{array}{cc} A & M\\ 0 & I_{q} \end{array}\right],\\ \bar{B}=\left[\begin{array}{c} B\\ 0 \end{array}\right],\\ \bar{C}={\left[\begin{array}{c} C\\ N \end{array}\right]}^{T},\\ \bar{E_{a}}={\left[\begin{array}{c} E_{a}\\ 0 \end{array}\right]}^{T},\\ G={\left[\begin{array}{c} 0\\ I_{q} \end{array}\right]}^{T}. \end{array}$$

The following augmented system can be established

(28) $$\begin{array}{c} \left\{\begin{array}{c} z\left(k+1\right)=Rz\left(k\right)+Su\left(k\right)+\left(L_{1}+L_{2}\right)y\left(k\right),\\ \hat{\bar{x}}\left(k\right)=z\left(k\right)+Ty\left(k\right), \end{array}\right. \end{array}$$

where *z* represents the state vector of the dynamic system equation (26); *R*, *S*, *L*_1_, *L*_2_ and *T* are the gain matrices with appropriate dimensions. The estimation error can be defined as $e\left(k\right)=\bar{x}\left(k\right)-\hat{\bar{x}}\left(k\right)$.

The derivative of the estimation error can be calculated as

(29) $$\begin{array}{c} e\left(k+1\right)=\left(I-T\bar{C}\right)\bar{x}\left(k+1\right)-z\left(k+1\right)-TE_{s}\omega_{s}\left(k\right)\\ =\left[\left(I-T\bar{C}\right)\bar{A}-L_{1}\bar{C}\right]e\left(k\right)+\left[\left(I-T\bar{C}\right)\bar{A}-L_{1}\bar{C}-R\right]z\left(k\right)\\ +\left[\left(I-T\bar{C}\right)\bar{B}-S\right]u_{k}+\left[\left(\left(I-T\bar{C}\right)\bar{A}-L_{1}\bar{C}\right)T-L_{2}\right]y\left(k\right)\\ +\left(I-T\bar{C}\right)\bar{E_{a}}\omega_{a}\left(k\right)+\left(I-T\bar{C}\right)Gm^{d}\left(k\right)-L_{1}E_{s}\omega_{s}\left(k\right)-TE_{s}\omega_{s}\left(k+1\right). \end{array}$$

If the following relationships can be held:

(30) $$\begin{array}{c} \left(I-T\bar{C}\right)\bar{E_{a}}=0,\\ \left(I-T\bar{C}\right)\bar{A}-L_{1}\bar{C}=R,\\ \left(I-T\bar{C}\right)\bar{B}=S,\\ RT=L_{2}. \end{array}$$

The derivative of the estimation error can be expressed as

(31) $$\begin{array}{c} e\left(k+1\right)=\text{Re}\left(k\right)+\left(I-T\bar{C}\right)Gm^{d}\left(k\right)-L_{1}E_{s}\omega_{s}\left(k\right)-TE_{s}\omega_{s}\left(k+1\right). \end{array}$$

The proof of the necessary conditions for the existence of the observer for the augmented system (26) can be found in [33] and omitted in here.

**Theorem 2 .**

For the augmented system 23, there exists a robust observer in the form of equation (24) such that ${\left\|e\left(k\right)\right\|}_{l_{2}}\leq \sqrt{2}r{\left\|\gamma \left(k\right)\right\|}_{l_{2}}$ where $\gamma \left(k\right)={\left[\begin{array}{cc} m^{d}\left(k\right) & \omega_{s}\left(k\right) \end{array}\right]}^{T}$, if there exists a positive definite matrix *P* and matrix *Q*, such that

(32) $$\begin{array}{c} \left[\begin{array}{cccc} -P+I_{\bar{n}} & * & * & *\\ 0_{l_{\gamma }\times \bar{n}} & -r^{2}I_{l_{\gamma }} & * & *\\ 0_{l_{\gamma }\times \bar{n}} & 0_{l_{\gamma }\times l_{\gamma }} & -r^{2}I_{l_{\gamma }} & *\\ PA_{1}-Q\bar{C} & PV_{1}-QV_{2} & P{\bar{V}}_{2} & -P \end{array}\right]<0, \end{array}$$

where $A_{1}=\left(I-T\bar{C}\right)\bar{A}$, *Q*=*PL*_1_, $V_{1}=\left[\left(I-T\bar{C}\right)G0_{\bar{n}\times l_{n}}\right]$, *V*_2_=[0_*p*×*q*_*E*_*s*_], and ${\bar{V}}_{2}=-TV_{2}$.

**Proof**

Proof. Take the following Lyapunov function candidate for system (30)

(33) $$\begin{array}{c} V\left(k\right)=e^{T}\left(k\right)Pe\left(k\right), \end{array}$$

one has

(34) $$\begin{array}{c} \Delta V\left(k\right)=V\left(k+1\right)-V\left(k\right)\\ ={\left[\begin{array}{c} e\left(k\right)\\ \gamma \left(k\right)\\ \gamma \left(k+1\right) \end{array}\right]}^{T}\left(\left[\begin{array}{c} R\\ V_{1}-L_{1}V_{2}\\ {\bar{V}}_{2} \end{array}\right]P{\left[\begin{array}{c} R\\ V_{1}-L_{1}V_{2}\\ {\bar{V}}_{2} \end{array}\right]}^{T}+\left[\begin{array}{cc} -P & 0\\ 0 & 0 \end{array}\right]\right)\left[\begin{array}{c} e\left(k\right)\\ \gamma \left(k\right)\\ \gamma \left(k+1\right) \end{array}\right]. \end{array}$$

If *γ*(*k*)=0, from equations (32) and (34) one has Δ*V*(*k*) < 0. The error dynamic is asymptotically stable.

Let

(35) $$\begin{array}{c} \Gamma =\sum_{k=0}^{\infty }\left(\Delta V\left(k\right)+e^{T}\left(k\right)e\left(k\right)-r^{2}\gamma^{T}\left(k\right)\gamma \left(k\right)-r^{2}\gamma^{T}\left(k+1\right)\gamma \left(k+1\right)\right). \end{array}$$

We can derive

(36) $$\begin{array}{c} \Gamma =\sum_{k=0}^{\infty }{\left[\begin{array}{c} e\left(k\right)\\ \gamma \left(k\right)\\ \gamma \left(k+1\right) \end{array}\right]}^{T}\left[\left(\left[\begin{array}{c} R\\ V_{1}-L_{1}V_{2}\\ {\bar{V}}_{2} \end{array}\right]P\right)P^{-1}\right.\left.\left(P\left[\begin{array}{c} R\\ V_{1}-L_{1}V_{2}\\ {\bar{V}}_{2} \end{array}\right]\right)+\left[\begin{array}{cc} -P+I & 0\\ 0 & -r^{2}I \end{array}\right]\right]\left[\begin{array}{c} e\left(k\right)\\ \gamma \left(k\right)\\ \gamma \left(k+1\right) \end{array}\right]. \end{array}$$

Based on equations (32) and (36), we can derive

(37) $$\begin{array}{c} \sum_{k=0}^{\infty }\left(e^{T}\left(k\right)e\left(k\right)-r^{2}\gamma^{T}\left(k\right)\gamma \left(k\right)-r^{2}\gamma^{T}\left(k+1\right)\gamma \left(k+1\right)\right)+V\left(\infty \right)-V\left(0\right)<0. \end{array}$$

In view of the fact that *V*(*∞*) ≥ 0 and *V*(0)=0, we can derive

(38) $$\begin{array}{c} \sum_{k=0}^{\infty }e^{T}\left(k\right)e\left(k\right)-2r^{2}\gamma^{T}\left(k\right)\gamma \left(k\right)<0, \end{array}$$

which is equivalent to ${\left\|e\left(k\right)\right\|}_{l_{2}}\leq \sqrt{2}r{\left\|\gamma \left(k\right)\right\|}_{l_{2}}$. The proof is completed.

Based on the proposed observer, we can derive the observed data of the variables and the measured data of those in DDCA. For the defender, it is necessary to identify the similarities between the measured data and the observed data under normal situations and distinguish the differences under the compromised situations.

## 4. Detection Scheme against FDI Attack considering Dual Source Data

In this section, we study the attack detection scheme against FDI attacks based on the observed data of the variables and the measured data of those in DDCA. A relation-based detection network is proposed to extract the similarity of the dual source data. We design the machine-learning-based detection scheme based on the following considerations:

- The method of calculating dual source data vector similarity based on traditional Euclidean distance requires too much prior knowledge level of defenders. In this paper, we use an embedding module and a relation module to extract the similarity of the dual source data automatically.
- Traditional machine learning methods need the distance of data vector in feature space to identify, which means that large scale of training data set is needed. In this paper, we skip the learning of feature distance and directly learn the relationship between dual source data, so as to effectively reduce the demand for the size of data set.

As is shown in Figure 1, the detection network contains measured data set, observed data set, Embedding module, and relation module. The data in the observed data set can reflect the current real operating state of the DDCA system, and the data in the measured data set may be tampered with. As to the attack detection network, we identify the attack by comparing the observed data with measured data. The measured data set consists of the compromised data set and the normal data set. When the data for comparison comes from the compromised data set, the relationship between dual source data is strong similarity. When the data for comparison comes from the normal data set, the relationship between two dual data is weak similarity.

As to the datasets, the data vectors in each dataset consists of the time series data of target variables in DDCA, including the data of incremental cost and those of output power. The data vector in the measured data set is written as *d*_*m*_. The data vector in the observed data set is written as *d*_*o*_. The embedding module, which consists of full connect layers and rectified linear units (ReLUs), is used to extract the features of samples with a nonlinear function *ℰ*. Compared with the traditional manual feature extraction method, the feature extraction by full connect layers can reduce the prior knowledge requirements of attack detection network for attack features. Rectified linear units are used to improve the generalization ability of the embedding module. The feature vectors of measured data and observed data generated by the embedding module can be expressed as ℱ(*d*_*m*_) and ℱ(*d*_*o*_). To alleviate the over fitting problem of the embedding module, class prototype of each feature vector class is adopted. The prototype *𝒫*_*i*_^*m*^ of the measured data feature vectors and the prototype *𝒫*_*i*_^*o*^ of the observed data feature vectors can be expressed as

(39) $$\begin{array}{c} P_{i}^{m}=\frac{1}{N_{i}^{m}}\sum_{j=1}^{N_{i}^{m}}ℱ\left(d_{m}\right),\\ P_{i}^{o}=\frac{1}{N_{i}^{o}}\sum_{j=1}^{N_{i}^{o}}ℱ\left(d_{o}\right). \end{array}$$

We can derive the class feature vector *𝒞*(*𝒫*_*i*_^*m*^, *𝒫*_*i*_^*o*^) by concatenating the prototypes in depth dimension. The relation module is used to extract the similarity between the concatenations with a nonlinear relation function ℛ. The similarity *𝒮* can be written as

(40) $$\begin{array}{c} S=ℛ\left(C\left(P_{i}^{m},P_{i}^{o}\right)\right). \end{array}$$

To train the attack detection model, mean square error (MSE) is used as the objective function *L*_*m*_.

(41) $$\begin{array}{c} L_{m}=\left\{\begin{array}{c} \sum \sum {\left(S-1\right)}^{2},l_{m}=l_{o},\\ \sum \sum {\left(S-0\right)}^{2},l_{m}\neq l_{o}. \end{array}\right. \end{array}$$

If the measured data is compromised, then *l*_*m*_ ≠ *l*_*o*_ and *𝒮* is closed to 0. If the measured data is normal, then *l*_*m*_=*l*_*o*_ and *𝒮* is closed to 1.

Pseudocode for the proposed detection scheme is provided in Figure 2. First, input samples of variables of interest in DDCA as measured data set. Label the compromised data and the normal data. Then, use the proposed observer to observe the variables and form the observed data set. Then, obtain the feature vectors and prototype vectors in order with the help of the proposed module. Based on the relation feature vector concatenated by prototype vectors, calculate the similarity score using relation module. Based on the proposed objective function, optimize the model parameters with the stochastic gradient descent optimizer. After training the model, sample the incoming data, calculate the similarity and output the type of the test data.

## 5. Case Study

In this section, simulations are carried out to illustrate the effectiveness of the proposed observer and attack detection network of the variables in DDCA. The Barry Island electricity and heating networks is used as the tested system. The structure and parameters of the system can be found in [34].

### 5.1. Performance of the Observer for the Compromised System

In the DDCA system, the coefficient matrices are

(42) $$\begin{array}{c} A=\left[\begin{array}{cccc} 0.9988 & 0.0007 & 0.0006 & -0.0037\\ 0.0014 & 0.98 & -0.0012 & -0.0206\\ 0.001 & 0.0037 & 1.0467 & 9.5584\\ 0 & 0 & 0.0101 & 1.0234 \end{array}\right],\\ B=\left[\begin{array}{cc} 0.0052 & 0.0012\\ 0.0315 & -0.0755\\ -0.0582 & 0.0454\\ -0.0003 & 0.0002 \end{array}\right],\\ C=\left[\begin{array}{cccc} 0.45 & 0.32 & 0.12 & 0.11\\ 0.38 & 0.42 & 0.13 & 0.07\\ 0.27 & 0.31 & 0.33 & 0.09\\ 0.07 & 0.13 & 0.43 & 0.37 \end{array}\right]. \end{array}$$

The attack vector is $m\left(k\right)={\left[\begin{array}{cc} m_{1}\left(k\right) & m_{2}\left(k\right) \end{array}\right]}^{T}$, where

(43) $$\begin{array}{c} m_{1}\left(k\right)=\left\{\begin{array}{cc} 0, & k<60,\\ 0.05\left(k-60\right), & 60\leq k<100,\\ 2, & k\geq 100, \end{array}\right.\\ m_{2}\left(k\right)=\left\{\begin{array}{cc} 0, & k<60,\\ 1, & k\geq 60. \end{array}\right. \end{array}$$

First, we illustrate the performance of observer against false data injection attacks on incremental cost estimator. The attack target variable is *x*_*p*_^*P*^. Based on the method proposed in Section 1, the observed data of the variable *x*_*p*_^*P*^ can be obtained. The simulation result of the dual source data is shown in Figure 3. The observation error is shown in Figure 4. It can be learned that when the attack volume is a static value, the observed data can effectively track the measured data. When the attack volume changes, there is a certain observation error between the observed data and the measured data, because the changed attack volume is equivalent to the changing disturbance volume. The difference between the observed data and the measured data will be an important basis for the attack detection network to identify whether the system is compromised.

Then, the performance of observer against false data injection attacks on output power decision-maker is studied. The attack target variable is *y*_*p*_^*C*^. Based on the method proposed in Section 2, the observed data of the state variable *x*_*p*_^*C*^ in DDCA can be obtained. The simulation results are shown in Figures 5 and 6.

It can be learned that the FDI attacks on electric output power *y*_*p*_^*C*^ in the output power decision-maker makes the measured incremental cost data *x*_*p*_^*P*^ different from the observed ones. Compared with the FDI attacks on incremental cost estimator, the impact of FDI attacks on output power decision-maker can be reflected by the variables in incremental cost estimator.

To illustrate the performance of the proposed observer in situations of multiple modules being compromised, we analysis the simulation results considering the situation that *x*_*h*_^*C*^ and *y*_*h*_^*C*^ are compromised simultaneously. Based on the method proposed in Section 3, the observed data of the variable *x*_*h*_^*C*^ can be obtained. The simulation results are shown in Figures 7 and8. It can be learned that there are obvious differences between the measured data and the observed data. The difference of dual source data is affected by the attack volume, as well as the system noise, disturbance and delay. Therefore, it is necessary to identify whether the system is compromised based on the attack detection scheme.

### 5.2. Performance of the Observer for the Relation-Based Attack Detection Scheme

In this subsection, we evaluate the performance of the proposed attack detection scheme. In the embedding module, there are three full connect layers and rectified linear units. The batch size of the relation network is chosen as 20. In the measured data set, there are 500 normal sample data and 500 compromised data from the historical database. In the observed data set, 1000 observed data are generated based on the proposed method studied in Section B. The simulations are carried out on a personal computer with Intel processor core i7, cache 3.4 GHz, NVIDIA GTX 2060, and random-access memory (RAM) 32 GB.

To evaluate the performance of the relation-based attack detection scheme, the following metrics are used:

(1) Accuracy:
  (44) $$\begin{array}{c} MA=\frac{TP+TN}{TP+TN+FP+FN}, \end{array}$$
where *TP* represents the number of true positive detection results; *TN* represents the number of true negative detection results; *FP* represents the number of false positive detection results; *FN* represents the number of false negative detection results.
(2) The probability of detecting correctly:
  (45) $$\begin{array}{c} MD=\frac{TP}{TP+FN}. \end{array}$$
(3) Success ratio:
  (46) $$\begin{array}{c} MS=\frac{TP}{TP+FP}. \end{array}$$
(4) Probability of identifying normal cases:
  (47) $$\begin{array}{c} MI=\frac{TN}{TN+FP}. \end{array}$$
(5) Trade off between *M*_*dc*_ and *M*_*s*_:
  (48) $$\begin{array}{c} MF\left(T\right)=\frac{\left(1+T^{2}\right)\cdot M_{dc}\cdot M_{s}}{T^{2}\cdot M_{dc}+M_{s}}, \end{array}$$
where *𝒯* is the trade-off coefficient. Details about the performance metrics can be found in [31].

To illustrate the effectiveness of the proposed detection scheme, six methods are adopted for comparison: (1) The proposed relation-based attack detection scheme (ME1); (2) Attack detection scheme using relation network without prototype module (ME2); (3) Attack detection scheme using multi-layer perception (ME3); (4) Attack detection scheme using signal forecasting method (ME4); (5) Attack detection scheme using support vector machine (ME5); (6) Attack detection scheme using clustering artificial bee colony algorithm (ME6).

The simulation results are shown in Figure 9. Compared with other attack detection scheme, the attack detection scheme (ME1) proposed in this paper has better performance in each algorithm evaluation index, that is, the proposed detection scheme can effectively detect false data injection attacks on variables in DDCA. The better performance of the proposed attack detection scheme mainly comes from the fact that the relation-based attack detection network focuses on exploiting the differences between normal data and compromised data, while the other attack detection schemes focus on exploiting the features. If the common features of normal data and compromised data are learned by the other attack detection schemes, it will have a negative impact on the performance of the attack detection schemes.

### 5.3. Stability and Reliability of the Relation-Based Attack Detection Scheme

In order to further investigate the stability of the detection performance of the proposed attack detection scheme, the performance of the attack detection scheme with different proportion of training sets is studied: at an interval of 5%, samples with a proportion from 40% to 80% are selected as the training sets. The simulation results are shown in Figure 10. It can be seen that although the performance of the proposed attack detection scheme will decline with the sample size, and the performance of some training sample sizes is inferior to other schemes, its overall attack detection performance is basically in the first echelon, which verifies that the attack detection scheme still has excellent detection effect under the sample size discussed in this section.

Considering the insufficient samples of compromised data in practice, we further discuss the reliability and stability under different positive and negative sample ratios. In this section, the ratio of positive samples to negative samples is 1 : 1, 1 : 2, 1 : 5 and 1 : 10 respectively. The specific performance verification effect is shown in Figure 11. It can be learned that when the number of positive samples is smaller than the number of negative samples, the performance of the proposed attack detection scheme will decline to a certain extent, but the overall performance still has certain advantages over other detection schemes. The decline of detection performance is mainly due to the fact that the attack detection network can not fully learn the difference between positive and negative samples.

Considering that the detection scheme proposed in this paper depends on the real-time data of the sensors, we further study the impact of measurement noise and measurement delay on the attack detection performance in the process of collecting sensor data. We design two metrics, security noise and security delay, to evaluate the detection performance of the proposed attack detection method. Safe noise (delay) refers to the maximum noise (delay) that can be tolerated when the detection accuracy (MA) reaches a specified threshold.

Safe noise and safe delay considering different threshold of MA are in Table 1. It can be learned that the safe noise (delay) decreases with the increase of the threshold. It can be seen that when there are high requirements for the accuracy of the detection scheme, the data required by the detection scheme is also more ideal. Noise and delay have a significant impact on the detection effect. Correspondingly, if the requirements for detection performance are appropriately reduced, the proposed detection scheme has a certain tolerance to noise and delay. As a remedy, the defender should also consider using a variety of detection schemes to cross check the attack behavior, so as to improve the overall accuracy.

## 6. Conclusions and Discussions

### 6.1. Conclusions

In this article, false data injection attacks on distributed controller of electric-thermal integrated energy system and countermeasures are studied. Observers of variables in DDCA are designed to track the compromised data. The proposed observer can achieve the observation considering different attack targets in DDCA. Based on the observed data and the measured data, we proposed a relation-based attack detection scheme to identify the false data injection attacks.

The simulation results show that the attack detection scheme has better performance than the current mainstream scheme under multiple evaluation indexes. The better detection performance of the proposed scheme is attributed to its direct judgment of the difference between normal data pairs and compromised data pairs, which reduces the learning of other unnecessary or incorrect features. For the stability of the proposed scheme, compared with other schemes, the proposed scheme can maintain better detection performance with less proportion of training sets.

Therefore, we believe that the proposed attack detection scheme can achieve good performance against FDI attacks on ETIES.

### 6.2. Discussions

It can be seen that the limitation of the proposed method used in this paper is that it requires real-time data of the system, which makes the defender have a certain dependence on the real-time sensor communication network. As to practical implementation, the challenge is how to deal with the large-scale destruction of more sensors by attackers. In such a scenario, the trusted data available in this paper will be reduced, and the ability to identify attacks will be reduced.

A possible mitigation approach is to stop using the real-time data obtained by the sensors of the system. As an alternative, the defender can use the system model and historical data to generate prediction data for real-time data, and use the predicted data combined with the algorithm proposed in this paper to identify cyber attacks. It can be seen that this research idea further reduces the dependence on real-time sensors, thereby reducing the uncertainty under large-scale attacks.

## Figures and Tables

**Figure 1:** The relation network for FDI attack detection.

**Figure 2:** Pseudocode for the proposed detection scheme.

**Figure 3:** Dual source data of variable *x*_*p*_^*P*^ under FDI attacks on incremental cost estimator.

**Figure 4:** Observation error of variable *x*_*p*_^*P*^ under FDI attacks on incremental cost estimator.

**Figure 5:** Dual source data of variable *x*_*p*_^*C*^ under FDI attacks on output power decision-maker.

**Figure 6:** Observation error of variable *x*_*p*_^*C*^ under FDI attacks on output power decision-maker.

**Figure 7:** Dual source data of variable *x*_*h*_^*C*^ under FDI attacks on multiple modules.

**Figure 8:** Observation error of variable *x*_*h*_^*C*^ under FDI attacks on multiple modules.

**Figure 9:** Performance of different attack detection method.

**Figure 10:** Performance of detection schemes considering different training set proportion. (a) MA. (b) MD. (c). MS. (d) MI.

**Figure 11:** Performance of detection schemes considering different ratio of positive samples to negative samples. (a) MA. (b) MS. (c) MS. (d) MI.

**Table 1:** Safe noise and delay considering different threshold of detection accuracy.

Threshold of MA	75%	80%	85%	90%
Safe noise	15.2 dB	11.3 dB	9.8 dB	4.4 dB
Safe delay	7.2 s	5.7 s	2.9 s	2.1 s

## Data Availability

The data used to support the findings of this study are available from the corresponding author upon request.

## References

[1] Qian A., Ran H. (2018). Key technologies and challenges for multi-energy complementarity and optimization of integrated energy system. *Automation of Electric Power Systems*.

[2] Li J., Fang J., Zeng Q., Chen Z. (2016). Optimal operation of the integrated electrical and heating systems to accommodate the intermittent renewable sources. *Applied Energy*.

[3] Li J., Zhu M., Huang Y. (2019). Classification and location scheme selection of coupling components in integrated electrical and heating systems with renewable energy. *CSEE Journal of Power and Energy Systems*.

[4] Ding Y., Jiang Y., Song Y. (2016). Review of risk assessment for energy internet, part i: physical level. *Proceedings of the CSEE*.

[5] Yibao J., Yonghua S., Yi D., Chuangxin G., Wende J. (2016). Review of risk assessment for energy internet part t ii: information and market level. *Proceedings of the CSEE*.

[6] Mahmoud M. S., Khalid H. M., Hamdan M. M. (2021). *Cyberphysical Infrastructures in Power Systems: Architectures and Vulnerabilities*.

[7] He W., Xu W., Ge X., Han Q.-L., Du W., Qian F. (2022). Secure control of multi-agent systems against malicious attacks: a brief survey. *IEEE Transactions on Industrial Informatics*.

[8] Miao Y., Chen C., Pan L., Han Q.-L., Zhang J., Xiang Y. (2022). Machine learning–based cyber attacks targeting on controlled information: a survey. *ACM Computing Surveys*.

[9] Khalid H. M., Muyeen S. M., Peng J. C.-H. (2020). Cyber-attacks in a looped energy-water nexus: an inoculated sub-observer-based approach. *IEEE Systems Journal*.

[10] Chen C., Wang Y., Cui M. (2022). Data-driven detection of stealthy false data injection attack against power system state estimation. *IEEE Transactions on Industrial Informatics*.

[11] Liu Y., Ning P., Reiter M. K. (2011). False data injection attacks against state estimation in electric power grids. *ACM Transactions on Information and System Security*.

[12] Molnár M., Vokony I. Impact analysis of false data injection attacks on distribution system state estimation.

[13] Khalid H. M., Peng J. C.-H. (2016). A bayesian algorithm to enhance the resilience of wams applications against cyber attacks. *IEEE Transactions on Smart Grid*.

[14] Khalid H. M., Peng C. H. (2017). Immunity toward data-injection attacks using multisensor track fusion-based model prediction. *IEEE Transactions on Smart Grid*.

[15] Sandberg H., Teixeira A., Johansson K. H. On security indices for state estimators in power networks.

[16] Sou K. C., Sandberg H., Johansson K. H. Electric power network security analysis via minimum cut relaxation.

[17] Dán G., Sandberg H. Stealth attacks and protection schemes for state estimators in power systems.

[18] Kim T. T., Poor H. V. (2011). Strategic protection against data injection attacks on power grids. *IEEE Transactions on Smart Grid*.

[19] Kosut O., Jia L., Thomas R. J., Tong L. Malicious data attacks on smart grid state estimation: attack strategies and countermeasures.

[20] Sou K. C., Sandberg H., Johansson K. H. (2012). Computing critical *k* -tuples in power networks. *IEEE Transactions on Power Systems*.

[21] Mrabet Z. E., Kaabouch N., Ghazi H. E., Ghazi H. E. (2018). Cyber-security in smart grid: survey and challenges. *Computers & Electrical Engineering*.

[22] Kim J., Tong L. (2013). On topology attack of a smart grid: undetectable attacks and countermeasures. *IEEE Journal on Selected Areas in Communications*.

[23] Deb D., Chakraborty S. R., Lagineni M., Singh K. (2020). Security analysis of MITM attack on SCADA network. *Machine Learning, Image Processing, Network Security and Data Sciences*.

[24] Kim J., Tong L., Thomas R. J. (2014). Data framing attack on state estimation. *IEEE Journal on Selected Areas in Communications*.

[25] Liu X., Zhu P., Zhang Y., Chen K. (2015). A collaborative intrusion detection mechanism against false data injection attack in advanced metering infrastructure. *IEEE Transactions on Smart Grid*.

[26] Li B., Lu R., Choo K.-K. R., Wang W., Luo S. (2019). On reliability analysis of smart grids under topology attacks: a stochastic petri net approach. *ACM Transactions on Cyber-Physical Systems*.

[27] Chen C., Zhang K., Yuan K., Zhu L., Qian M. (2018). Novel detection scheme design considering cyber attacks on load frequency control. *IEEE Transactions on Industrial Informatics*.

[28] Xun P., Zhu P., Zhang Z., Cui P., Xiong Y. (2018). Detectors on edge nodes against false data injection on transmission lines of smart grid. *Electronics*.

[29] Ahmed S., Lee Y., Hyun S.-H., Koo I. (2019). Unsupervised machine learning-based detection of covert data integrity assault in smart grid networks utilizing isolation forest. *IEEE Transactions on Information Forensics and Security*.

[30] Bi W., Zhang K., Li Y., Yuan K., Wang Y. (2019). Detection scheme against cyber-physical attacks on load frequency control based on dynamic characteristics analysis. *IEEE Systems Journal*.

[31] Cui M., Wang J., Yue M. (2019). Machine learning-based anomaly detection for load forecasting under cyberattacks. *IEEE Transactions on Smart Grid*.

[32] Sun Q., Fan R., Li Y., Huang B., Ma D. (2019). A distributed double-consensus algorithm for residential we-energy. *IEEE Transactions on Industrial Informatics*.

[33] Gao Z., Liu X., Chen M. Z. (2015). Unknown input observer-based robust fault estimation for systems corrupted by partially decoupled disturbances. *IEEE Transactions on Industrial Electronics*.

[34] Liu X., Wu J., Jenkins N., Bagdanavicius A. (2016). Combined analysis of electricity and heat networks. *Applied Energy*.

